The article "Immunoinformatic strategy for developing multi-epitope subunit vaccine against Helicobacter pylori" was retracted in 2025. Reasons: compromised peer review; concerns about the authorship.

# Immunoinformatic strategy for developing multi-epitope subunit vaccine against *Helicobacter pylori*

**DOI:** 10.1371/journal.pone.0318750

**Published:** 2025-02-07

**Authors:** Md. Nahian, Md. Rasel Khan, Fabiha Rahman, Hossain Mohammed Reza, Imren Bayil, Tanjum Ahmed Nodee, Tabassum Basher, Mostafizur Rahaman Sany, Rabeya Najnin Munmun, S. M. Ariful Habib, Lincon Mazumder, Mrityunjoy Acharjee

**Affiliations:** 1 Department of Microbiology, Jagannath University, Dhaka, Bangladesh; 2 Faculty of Life and Health Sciences, School of Pharmacy and Pharmaceutical Sciences, Ulster University, Coleraine, Northern Ireland; 3 Department of Bioinformatics and Computational Biology, Gaziantep University, Gaziantep, Turkey; 4 Department of Microbiology, Stamford University Bangladesh, Dhaka, Bangladesh; University of Chittagong, BANGLADESH

## Abstract

*Helicobacter pylori* is a gram-negative bacterium that persistently infects the human stomach, leading to peptic ulcers, gastritis, and an increased risk of gastric cancer. The extremophilic characteristics of this bacterium make it resistant to current drug treatments, and there are no licensed vaccines available against *H*. *pylori*. Computational approaches offer a viable alternative for designing antigenic, stable, and safe vaccines to control infections caused by this pathogen. In this study, we employed an immunoinformatic strategy to design a set of candidate multi-epitope subunit vaccines by combining the most potent B and T cell epitopes from three targeted antigenic proteins (BabA, CagA, and VacA). Out of the 12 hypothetical vaccines generated, two (HP_VaX_V1 and HP_VaX_V2) were found to be strongly immunogenic, non-allergenic, and structurally stable. The proposed vaccine candidates were evaluated based on population coverage, molecular docking, immune simulations, codon adaptation, secondary mRNA structure, and *in silico* cloning. The vaccine candidates exhibited antigenic scores of 1.19 and 1.01, with 93.5% and 90.4% of the most rama-favored regions, respectively. HP_VaX_V1 and HP_VaX_V2 exhibited the strongest binding affinity towards TLR-7 and TLR-8, as determined by molecular docking simulations (ΔG = −20.3 and −20.9, respectively). Afterward, multi-scale normal mode analysis simulation revealed the structural flexibility and stability of vaccine candidates. Additionally, immune simulations showed elevated levels of cell-mediated immunity, while repeated exposure simulations indicated rapid antigen clearance. Finally, *in silico* cloning was performed using the expression vector pET28a (+) with optimized restriction sites to develop a viable strategy for large-scale production of the chosen vaccine constructs. These analyses suggest that the proposed vaccines may elicit potent immune responses against *H*. *pylori*, but laboratory validation is needed to verify their safety and immunogenicity.

The article "Immunoinformatic strategy for developing multi-epitope subunit vaccine against Helicobacter pylori" was retracted in 2025. Reasons: compromised peer review; concerns about the authorship.

## Introduction

*Helicobacter pylori* is a spiral-shaped, microaerophilic, gram-negative bacterium that infects almost half of the global population, establishing its position as one of the most prevalent pathogens worldwide [1]. The International Agency for Research on Cancer (IARC) has classified *H*.*pyloryi* as a definite (class I) carcinogen due to its strong association with gastric malignancies [2]. This microorganism exhibits remarkable adaptability, enabling its survival in the highly acidic environment of the human stomach [3]. Transmission primarily occurs via direct contact with contaminated feces, saliva, vomit, food, or water from an infected individual [4]. Colonization typically begins during childhood, around the age of ten, and often persists throughout life [4]. Although often asymptomatic, infection can cause inflammation of the stomach lining, leading to severe illnesses such as peptic ulcers, stomach cancer, gastric cancer, chronic gastritis, or lymphoma [4, 5]. The occurrence of *H*. *pylori* in Western countries varies from 30% to 50%, but in developing nations, it is as high as 85% to 95% [6]. In Southern Asia, countries like India and Pakistan report the highest prevalence rates, at 63.5% and 81%, respectively [6].

The standard treatment for *H*. *pylori* infection involves a multi-drug regimen combining proton pump inhibitors (PPIs) and antibiotics for at least a week. While this regimen is generally effective, it is associated with several limitations. Firstly, it requires patients to take a high pill burden, particularly antibiotics, which can lead to dissatisfaction and, more importantly, contribute to the rise of antibiotic resistance [7]. This growing resistance is a significant global concern, hindering eradication efforts. Studies in China highlight concerning resistance rates to commonly used antibiotics like Metronidazole (60–70%), Clarithromycin (20–38%), and Levofloxacin (30–38%) [7]. Secondly, prolonged antibiotic use can disrupt the delicate balance of gut microbiota, potentially leading to other gastrointestinal or physiological problems [8]. Furthermore, antibiotic therapy offers no protection against reinfection. Despite extensive global research and the development of several potential vaccines, there is currently no approved vaccine to prevent *H*. *pylori* infection. So far, only one candidate has made it to phase III clinical trials [9, 10]. This underscores the urgent need for alternative strategies, such as safe and effective vaccines, to prevent and control *H*. *pylori* infection. A successful vaccine could offer a sustainable solution to this global public health challenge.

The article "Immunoinformatic strategy for developing multi-epitope subunit vaccine against Helicobacter pylori" was retracted in 2025. Reasons: compromised peer review; concerns about the authorship.

An epitope-based strategy is a novel and innovative approach that has seen significant advancements in recent years. This computational approach offers a time- and cost-efficient method to identify potential vaccine targets (epitopes) within specific proteins [11]. Unlike traditional vaccines targeting specific bacterial strains, epitope-based vaccines can provide broader protection [12]. The increasing availability of biological databases and advancements in next-generation sequencing have fueled the popularity of this technique for vaccine development [13]. By pinpointing optimal ligands for human leukocyte antigens (HLAs), this method allows for the precise identification of T-cell epitopes, which are crucial for eliciting effective immune responses [14]. Driven by this potential, researchers have extensively studied various *H*. *pylori* virulence proteins in the pursuit of a vaccine that combats stomach cancer and lymphoma [1]. Proteins that exhibited required immunogenic qualities for disease prevention in previous animal studies or computational analyses were prioritized as prime epitope candidates [15–18]. Among these, the cytotoxin-associated antigen (CagA) protein is seen as a possible target for vaccination as it is highly conserved among *H*. *pylori* strains [19]. Previous research has confirmed CagA as a primary focus of the immune response in susceptible BALB/c mice [20]. CagA plays a key role in carcinogenesis, synthesized by the Cag pathogenicity island in addition to a type 4 secretion system (T4SS). It is typically linked to a higher occurrence of inflammatory reactions and causes more extensive damage to the stomach mucosa [21]. Another potential vaccine candidate is the vacuolating cytotoxin gene A (VacA), which significantly contributes to the development of *H*. *pylori*-related conditions like stomach cancer and peptic ulcers [22–24]. By facilitating colonization and persistence within the human gastric mucosa, VacA can directly harm the stomach lining [25]. According to the study by Salama et al. (2001), a VacA-producing *H*. *pylori* strain had a significant advantage in colonizing the mouse stomach compared to a similar strain without the vacA gene [26]. Therefore, targeting VacA for vaccine development could potentially prevent these harmful effects and provide a means of protection against *H*. *pylori* infections [22]. Additionally, BabA is another prominent virulent protein of *H*. *pylori* on the external membrane of the bacteria that allows it to attach to the Lewis^b^ blood group antigens in the mucosal lining, thus helping the bacteria establish themselves and influencing their population size [27]. BabA and Le^b^ antigen binding may be essential for the type four secretion system (T4SS) to activate, which in turn causes the stomach to become more inflamed [28]. Research by Bugaytsova et al. (2023) demonstrated that mucosal immunization with the BabA protein in rhesus macaques elicited antibodies capable of preventing infection [29]. A mouse model showed that vaccination with BabA protein significantly decreased gastric inflammation and provided complete protection against *H*. *pylori*-related gastric cancer [29]. Research by Gordon (2000) found that in duodenal ulcer cases, 100% of patients were positive for BabA, CagA, and VacA, compared to 74% of patients with gastric cancer, 35% with MALT lymphoma, and 43% with antral gastritis [30]. Therefore, combining these key virulence factors (CagA, VacA, and BabA) simultaneously through a multi-epitope-based vaccination strategy could potentially elicit a broader and more robust immune response, leading to a more effective preventative measure against *H*. *pylori* infection and its associated gastric diseases. Additionally, by including multiple proteins in the vaccine formulation, the efficacy of the vaccine could be enhanced by reducing the likelihood of immune escape due to mutations in a single protein target.

The article "Immunoinformatic strategy for developing multi-epitope subunit vaccine against Helicobacter pylori" was retracted in 2025. Reasons: compromised peer review; concerns about the authorship.

The present study aims to design a broadly protective vaccine against *H*. *pylori* by incorporating epitopes from CagA, VacA, and BabA proteins using various immunoinformatic platforms. Immunogenic epitopes will be identified and combined to create a multi-epitope vaccine candidate, which will then be evaluated computationally for its physicochemical, chemical, and immunological properties.

## Methods

A schematic overview of the experimental methodologies employed in this study is presented in Fig 1.

**Fig 1:** Schematic representation of the workflow for the design of a multi-epitope vaccine against *Helicobacter pylori*.

### Sequence retrieval and target protein selection

The complete amino acid sequences of the *Helicobacter pylori* proteins CagA (WP_212850760.1), VacA (WP_202139098.1), and BabA (WP_187888179.1) were retrieved from the NCBI Protein database (https://www.ncbi.nlm.nih.gov/protein) [31]. The antigenicity of these proteins was evaluated using the VaxiJen 2.0 web server (https://www.ddg-pharmfac.net/vaxijen/VaxiJen/VaxiJen.html) with a threshold value of 0.4 [32]. VaxiJen applies an alignment-independent approach based on the physicochemical properties of proteins to predict their antigenicity [32]. The AllerTOP 2.0 server (https://www.ddg-pharmfac.net/AllerTOP/) was employed to evaluate the allergenicity of proteins based on antigenicity scores obtained from VaxiJen [33]. AllerTOP employs a machine learning algorithm based on an auto-cross-covariance (ACC) transformation of protein sequences into numerical vectors to classify allergens and non-allergens [33]. Subsequently, surface localization of the selected proteins was determined using the TMHMM 2.0 web server (https://services.healthtech.dtu.dk/service.php?TMHMM-2.0), which uses a hidden Markov model to predict the transmembrane helices and extracellular portions of the proteins [34]. Only the extracellular portions of CagA, VacA, and BabA were selected as potential vaccine targets in this study.

The article "Immunoinformatic strategy for developing multi-epitope subunit vaccine against Helicobacter pylori" was retracted in 2025. Reasons: compromised peer review; concerns about the authorship.

### Identification and filtration of Linear B lymphocyte (LBL), MHC I (CTL) and MHC II (HTL) epitopes

The ABCpred server (http://crdd.osdd.net/raghava/abcpred/) was utilized to identify potential linear B-cell epitopes likely to stimulate antibody production [35]. This server employs a recurrent neural network (RNN) architecture incorporating sparse and Blosum encodings, along with hidden Markov model inputs to predict epitopes within antigen sequences [35]. The minimum length required for LBL epitope prediction was 16 amino acids, with a threshold score of 0.51. The IEDB "MHC-I Binding Predictions" tool (http://tools.iedb.org/mhci/) was employed using the ANN 4.0 approach to predict MHC class I (CTL) epitopes [36]. This approach leverages advanced sequence-encoding schemes to improve the accuracy of T-cell epitope prediction by effectively capturing complex sequence relationships [37]. A broadly distributed set of Class I HLA alleles encompassing over 97% of the population was selected to optimize prediction coverage. The output was ranked by "Predicted IC50" values, with lower values indicating stronger binding between epitopes and alleles [38]. The NN-align 2.3 prediction algorithm, available through the IEDB MHC-II Binding Predictions web tool (http://tools.iedb.org/mhcii/), was utilized to predict MHC class II (HTL) epitopes [39]. This algorithm forecasts MHC class II epitopes by identifying binding cores and affinities, addressing data biases, and incorporating flanking residue information to improve predictive accuracy. The IEDB-recommended reference panel of 27 Class II HLA alleles, which provides coverage for 99% of the global population, was utilized for the analysis. The length of the epitope was defined as 15 amino acids. The prediction outputs for all HTL epitopes were chosen based on the "Adjacent rank" which is the percentile rank of a peptide’s binding affinity relative to a group of reference peptides. A lower percentile rank indicates a stronger predicted binding affinity and a higher likelihood of the peptide functioning as an epitope [40].

The article "Immunoinformatic strategy for developing multi-epitope subunit vaccine against Helicobacter pylori" was retracted in 2025. Reasons: compromised peer review; concerns about the authorship.

To refine the selection, the predicted LBL, CTL, and HTL epitopes were subjected to additional analysis. Toxicity was assessed using ToxinPred (http://crdd.osdd.net/raghava/toxinpred/) [41], antigenicity was assessed with Vaxijen 2.0 [32], and allergenicity was determined using AllerTOP v.2.0 (https://www.ddg-pharmfac.net/AllerTOP/method.html) [33]. Homology analysis was conducted using the NCBI protein BLAST tool to verify that the predicted epitopes were non-homologous to human proteins. E-values exceeding 0.0578 were considered indicative of non-homology, ensuring specificity in epitope selection [42, 43]. HTL epitopes were further screened for their potential to induce cytokine responses using IFNepitope (http://crdd.osdd.net/raghava/ifnepitope/) for interferon-gamma, IL4pred (https://webs.iiitd.edu.in/raghava/il4pred/design.php) for interleukin-4, and IL-10Pred (http://crdd.osdd.net/raghava/IL-10pred/) for interleukin-10. These servers rely on machine learning-based models trained on experimentally verified data to predict the likelihood of cytokine induction [44–46].

### Docking of the epitopes

Molecular docking was utilized to identify the binding affinity, analyze the interaction between CTL and HTL epitopes with their respective MHC alleles, evaluate structural compatibility, and predict the immune response to the epitopes [47]. The docking simulations required 3D structures of the peptide epitopes and the MHC alleles. The PEP-FOLD server (https://bioserv.rpbs.univ-paris-diderot.fr/services/PEP-FOLD/) was employed to predict the three-dimensional structures of the high-scoring epitopes [48]. PEP-FOLD applies a de novo approach that uses structural alphabet-based representations of amino acid sequences and molecular dynamics simulations to generate reliable 3D conformations for short peptides [48]. The 3D structures of MHC alleles were retrieved from the RCSB Protein Data Bank (RCSB PDB) (https://www.rcsb.org/) [49]. Cluspro (https://cluspro.bu.edu/publications.php) was then employed to perform the molecular docking simulations. ClusPro operates using a rigid-body docking algorithm that first generates numerous possible docking conformations (decoys) and then ranks them by clustering based on energy minimization, identifying the most stable binding interactions [50]. BIOVIA Discovery Studio Visualizer was utilized to visualize the docking data and eliminate unnecessary ligands [51]. Finally, the PRODIGY server (https://rascar.science.uu.nl/prodigy/) was employed to calculate the binding affinity of the epitope-allele complexes. PRODIGY estimates binding free energy using a combination of interfacial residue contact maps and machine learning models trained on experimental binding affinity data [52].

The article "Immunoinformatic strategy for developing multi-epitope subunit vaccine against Helicobacter pylori" was retracted in 2025. Reasons: compromised peer review; concerns about the authorship.

### Analysis of population coverage

The significant polymorphism of MHC molecules leads to considerable genetic diversity among individuals from different nations and ethnic groups. To ensure the wide applicability of the proposed vaccine, epitopes were selected based on their capacity to stimulate T cells across a broad range of MHC allele variations. The population coverage of the short-listed CTL and HTL epitopes was determined using the IEDB population coverage tool (http://tools.iedb.org/population/). This tool employs an algorithm that calculates the percentage of the population potentially covered by the selected epitopes, based on the prevalence of specific HLA alleles in different populations [53].

### Vaccine construction and analysis of physiochemical properties

Twelve distinct models targeting *H*. *pylori* infections were developed using various linkers, adjuvants, and epitope combinations. Vaccine constructs were categorized into two primary "design groups" according to the attachment patterns and positions of three selected virulence proteins: BabA, CagA, and VacA.

Design 1 involves interlinking CTL, HTL, and LBL epitopes using AAY, GPGPG, and KK linkers (S2A Fig). The AAY linker was selected for its capacity to enhance proteasomal cleavage, thereby improving MHC class I presentation and subsequent cytotoxic T-cell responses [54]. In addition to its immunological role, the AAY linker has been shown to significantly influence protein properties such as hydrophilicity, flexibility, and secondary structure [55, 56]. The GPGPG linker was incorporated to separate HTL epitopes, as it has been reported to enhance immune responses and improve vaccine efficacy [57]. Moreover, glycine-rich sequences such as GPGPG are known to increase the flexibility of linked proteins without adversely affecting their functionality [56]. The KK linker, composed of bi-lysine residues, was employed to connect epitopes due to its ability to targeted lysosomal proteases, facilitating antigen processing while preserving the independent immunoreactivity of the vaccine construct [58].

Design 2 organized the virulence proteins VacA, BabA, and CagA based on their native amino acid sequence positions and connected them using a GGGGS linker (S2B Fig). The GGGGS linker, a widely used flexible sequence in fusion protein design, contains polar amino acids such as serine or threonine and small, non-polar residues like glycine. These properties facilitate inter-domain interactions, stabilize protein folding, and improve overall structural flexibility [59]. Furthermore, the GGGGS linker allows the optimal spatial arrangement of functional domains, preserving the immunogenic characteristics of epitopes in subunit vaccine constructs [58].

The article "Immunoinformatic strategy for developing multi-epitope subunit vaccine against Helicobacter pylori" was retracted in 2025. Reasons: compromised peer review; concerns about the authorship.

Each design was further categorized into six models, incorporating different adjuvants, including Melittin (P01501) [60], beta-defensin (Q5U7J2) [61], ribosomal protein L7/L12 (P9WHE3.1) [62], and PADRE sequences [63]. The adjuvant and padre sequence were added to the vaccine construct using the alpha-helical EAAAK linker, which was specifically selected for its ability to improve solubility and enhance adjuvant activity [64].

Following the development process, these models were subsequently evaluated on multiple web servers to predict their distinctive properties. VaxiJen 2.0 was used to forecast the antigenicity of the constructs [32], while their allergenicity was predicted using AllerTOP [33]. ToxinPred was used to indicate the toxicity levels of the constructs [41], while SOLpro (https://scratch.proteomics.ics.uci.edu/) was utilized for solubility prediction [65]. Additionally, stability, thermostability, and hydrophobicity were predicted using ProtParam [66]. The instability and aliphatic indexes assessed the proteins’ thermostability and strength. The hydrophilicity of the antigenic protein was determined by calculating the grand average of hydropathicity (GRAVY) value.

### Prediction of the secondary and tertiary structure of constructed vaccine

The PSIPRED web program (http://bioinf.cs.ucl.ac.uk/psipred/) was used to predict and visualize the secondary structure of the vaccine constructs. PSIPRED employs a neural network-based algorithm trained on known protein structures to predict secondary structure elements, including helices, sheets, and coils, from amino acid sequences with high accuracy [67]. To validate these predictions, the SOPMA webtool (https://npsa-prabi.ibcp.fr/cgi-bin/npsa_automat.pl?page=/NPSA/npsa_sopma.html) was used. SOPMA applies an alignment-free statistical approach based on the GOR (Garnier-Osguthorpe-Robson) method to categorize the structural components into four conformations: Helix, Sheet, Turn, and Coil [68]. The Robetta server (https://robetta.bakerlab.org/) was used to analyze and forecast the 3D structure of the construct sequence. Robetta uses a hybrid modeling approach, combining comparative modeling for regions with homologous templates and de novo structure prediction for non-homologous regions. The server integrates sequence analysis, domain identification, and fragment-based assembly to generate accurate 3D models of protein constructs [69]. The resulting structural models were imported and visualized using the BIOVIA Discovery Studio Visualizer, which facilitated the detailed examination of molecular architecture and conformation [51].

The article "Immunoinformatic strategy for developing multi-epitope subunit vaccine against Helicobacter pylori" was retracted in 2025. Reasons: compromised peer review; concerns about the authorship.

### Vaccine construct refinement and validation

The GalaxyRefine web server (https://galaxy.seoklab.org/cgi-bin/submit.cgi?type=REFINE) was employed for structural refinement. GalaxyRefine enhances the 3D model by iteratively rebuilding side chains, performing energy minimization, and optimizing the hydrogen bonding network. It uses molecular dynamics simulations to improve the overall geometry and quality of the model [70]. The accuracy and reliability of the predicted structure were validated using the ProSA web tool (https://prosa.services.came.sbg.ac.at/prosa.php), which assesses the model’s overall quality through Z-score analysis. This score provides insights into the structural reliability of the model by comparing it with experimentally resolved protein structures available in the Protein Data Bank (PDB). A Z-score within the range of native proteins indicates that the model’s structural quality is consistent with known proteins of similar lengths, ensuring its suitability for downstream analyses [71]. Further validation of the stereochemical characteristics of the vaccine construct was conducted using the PROCHECK web-based program (https://www.ebi.ac.uk/thornton-srv/software/PROCHECK/). PROCHECK evaluates the backbone and side-chain dihedral angles of the model and generates a Ramachandran plot, which illustrates the percentage of residues in favorable, allowed, and disallowed regions [72].

### Disulfide modification for improved vaccine peptide structural integrity

Disulfide linkages increase the free energy of the denatured state and decrease conformational entropy, which improves protein stability. The incorporation of novel disulfide bonds has been acknowledged as a significant biotechnological approach to augment the thermal stability of inherently folded proteins. The Disulfide by Design 2 (DbD2) server (http://cptweb.cpt.wayne.edu/DbD2/) was employed to enhance the structural integrity of the intended vaccination by including disulfide linkages [73]. This server simulates the substitution of residues with cysteine and calculates key parameters such as the energy score and chi3 angle, which are critical for disulfide bond formation. In this study, residue pairs with an energy value of ≤2.2 and a chi3 dihedral angle within the range of -87° to +97° were considered suitable candidates for disulfide bond formation. These identified residues were computationally modified by replacing them with cysteine residues to introduce new disulfide linkages, thereby improving the structural stability of the vaccine [73].

The article "Immunoinformatic strategy for developing multi-epitope subunit vaccine against Helicobacter pylori" was retracted in 2025. Reasons: compromised peer review; concerns about the authorship.

### Mapping discontinuous B cell epitopes in the constructed vaccine

Discontinuous B-cell epitopes are regions within a protein’s 3D structure where non-contiguous amino acid residues come into spatial proximity to stimulate B-cell responses. To identify these epitopes in the constructed vaccine, the PDB files were analyzed using ElliPro server (http://tools.iedb.org/ellipro/). ElliPro predicts conformational epitopes based on a protein’s 3D structure using a geometrical method that approximates protein shape as an ellipsoid. Residues are clustered based on protrusion indices (PI), calculated by comparing the residue’s distance from the ellipsoid’s center to the average distance of all residues [74]. The utmost distance was set at 6 Å, while the lowest score was fixed at 0.5. ElliPro has an impressive AUC value of 0.732, making it one of the best tools available today for conformational epitope prediction [74].

### Molecular interactions with TLRs

To assess the immune activation potential of the constructed vaccine, molecular docking studies were conducted to evaluate its interactions with various Toll-like receptors (TLRs), including TLR2 (PDB ID: 6NIG), TLR3 (PDB ID: 7C76), TLR4 (PDB ID: 4G8A), TLR5 (PDB ID: 3J0A), TLR6 (PDB ID: 3A79), TLR7 (PDB ID: 5GMG), TLR8 (PDB ID: 6ZJZ), and TLR9 (PDB ID: 3WPF). The 3D structures of these TLRs were retrieved from the Protein Data Bank (https://www.rcsb.org/). Docking simulations were conducted using the ClusPro server (https://cluspro.bu.edu/login.php), which applies an energy-based filtering approach to determine optimal docking poses. ClusPro uses Fast Fourier Transform (FFT)-based rigid-body docking combined with electrostatic, desolvation, and van der Waals scoring to identify the best candidate vaccine-receptor complexes [50]. The binding affinities of the docked vaccine-TLR complexes were further calculated using the PRODIGY server (https://nestor.science.uu.nl/prodigy/), which predicts binding free energy (ΔG) based on interatomic contacts and chemical properties of the docking interface [52].

### Normal mode analysis

To evaluate the stability and molecular flexibility of the highest-affinity vaccine-receptor complexes, multi-scale normal mode analysis (NMA) was performed using the iMod web server (http://imods.chaconlab.org). This computational framework simulates the conformational motions of macromolecules, enabling the identification of key dynamic features such as hinge regions, flexibility patterns, and structural stability. The insights gained from this analysis are crucial for understanding the functional dynamics and interaction robustness of the complexes [75].

The article "Immunoinformatic strategy for developing multi-epitope subunit vaccine against Helicobacter pylori" was retracted in 2025. Reasons: compromised peer review; concerns about the authorship.

### Molecular dynamics simulation analyses

All-atom molecular dynamics (MD) simulations were carried out using the GROMACS software package version 2020 with the CHARMM36 force field for proteins [76, 77]. The CHARMM-GUI server was employed to generate the topology and force field parameters for the proteins of interest [78]. Each protein was placed in a truncated octahedral box, ensuring a minimum distance of 10 Å between the protein and the edge of the box, and solubilized using TIP3P water molecules. To neutralize the system, potassium cations were added, followed by the addition of Na⁺Cl⁻ ion pairs to achieve a physiological ionic concentration of 0.15 M. Electrostatic interactions were handled using the particle mesh Ewald (PME) method, with a real-space cutoff distance set at 10 Å [79]. The van der Waals interactions were calculated using a switching function within a range of 12–14 Å. The grid spacing for PME calculations was set to 1.2 Å, and computations were performed at every simulation step without employing a multiple-time-stepping strategy. Prior to production runs, the energy of the docked protein complexes was minimized using the CHARMM36 force field, ensuring the elimination of steric clashes and unfavorable geometries. The minimized systems underwent equilibration in two stages. Initially, the systems were equilibrated in the NVT ensemble at 310 K for 5,000 steps (10 ps), followed by equilibration in the NPT ensemble under a constant pressure of 1 bar. Production MD simulations were carried out for 100 ns with a time step of 2 fs (dt = 0.002 ps), corresponding to 50,000,000 steps in total [80, 81]. The LINCS algorithm was applied to constrain all hydrogen bonds, enabling the use of a 2 fs time step. Temperature was maintained at 310 K using the velocity-rescale thermostat, while pressure was controlled using the Parrinello-Rahman barostat. Post-simulation, trajectory analysis was performed using VMD (University of Illinois at Urbana-Champaign, Urbana, IL, USA) and QTGRACE after re-centering the system. This approach allowed for in-depth assessment of protein-ligand dynamics, structural stability, and conformational flexibility.

### Immune simulation

The vaccine candidates were analyzed using the C-IMMSIM website (https://kraken.iac.rm.cnr.it/C-IMMSIM/index.php) [82] to anticipate the cellular humoral and immunologic responses, cellular entities, and cytokine responses. C-IMMSIM is an agent-based *in silico* immune system simulator that models both the innate and adaptive immune responses based on a position-specific scoring matrix (PSSM) framework. The system simulates interactions among immune entities, including B cells, T cells, dendritic cells, and cytokines, in response to the provided antigen’s structure. For this study, the PDB files of the vaccine constructs were uploaded to the server, and the immune response was monitored over a simulated one-year period (equivalent to 350 days). The simulated steps were set to 1050, while all other parameters were retained at their default values. Three *in silico* injections were administered at defined time steps (1, 84, and 170) to mimic a vaccination schedule, corresponding to real-world intervals of 8 hours per time step. Notably, lipopolysaccharide (LPS) was excluded from the simulation, and a minimum interval of 28 days was maintained between each *in-silico* injection.

The article "Immunoinformatic strategy for developing multi-epitope subunit vaccine against Helicobacter pylori" was retracted in 2025. Reasons: compromised peer review; concerns about the authorship.

### *In Silico* strategies for vaccine expression and cloning

To enable efficient expression of the vaccine candidate, the amino acid sequence was first converted into a nucleotide sequence using the EMBOSS Back-Translate tool (https://www.ebi.ac.uk/Tools/st/emboss_backtranseq/). This tool generates all possible codon combinations for a given protein sequence by referencing a codon usage table specific to the target organism, thereby ensuring accurate back-translation [83]. The resulting nucleotide sequence was subsequently optimized for expression in human cells using the GenSmart Codon Optimization Tool (https://www.genscript.com/tools/gensmart-codon-optimization). This platform utilizes an advanced codon adaptation algorithm that maximizes translation efficiency by aligning the codon usage bias with the codon preferences of the host organism, thereby enhancing protein expression [84]. Additionally, during the optimization process, recognition sites for the restriction enzymes Eco53KI and BstZ17I were eliminated to prevent unintended cleavage during subsequent cloning steps. Following optimization, the GenScript Rare Codon Analysis Tool (https://www.genscript.com/tools/rare-codon-analysis) was utilized to assess the efficiency of codon usage [85]. Three essential metrics for optimized protein expression were analyzed: (1) codon adaptation index (CAI) to assess translation efficiency, (2) codon frequency distribution (CFD) to detect potential codon usage biases, and (3) GC content. Afterward, the thermodynamic stability of the vaccine’s mRNA secondary structure was predicted using the RNAfold webserver (http://rna.tbi.univie.ac.at/cgi-bin/RNAWebSuite/RNAfold.cgi). This tool calculates the minimum free energy (MFE) and generates the most stable mRNA secondary structure [86]. Following this analysis, the optimized construct was inserted into the pET-28a(+) plasmid vector. The pET-28a(+) plasmid was selected for its suitability for high-level protein expression in *E*. *coli*. It features a strong T7 promoter for efficient transcription, an N-terminal His-tag to facilitate purification, and a versatile multiple cloning site (MCS) compatible with the vaccine construct [87]. Additionally, its kanamycin resistance marker ensures efficient selection, and its optimization for *E*. *coli* makes it an ideal choice for cost-effective and reliable recombinant protein production [87]. The cloning process was performed using SnapGene software, a widely recognized tool for molecular cloning simulations. Restriction enzyme recognition sites for Eco53KI and BstZ17I were strategically introduced at the 5′ and 3′ ends of the sequence to ensure precise insertion into the plasmid.

The article "Immunoinformatic strategy for developing multi-epitope subunit vaccine against Helicobacter pylori" was retracted in 2025. Reasons: compromised peer review; concerns about the authorship.

## Results

### Selection of target PROTEINS for vaccine design

The antigenicity analysis performed using Vaxijen 2.0 demonstrated that all three target proteins, CagA, VacA, and BabA, achieved scores exceeding the predefined threshold of 0.4, with values of 0.4939, 0.5935, and 0.4835, respectively. These results indicate a strong antigenic potential. Subsequently, AllerTOP v.2.0 confirmed that these candidate vaccine targets are non-allergenic. To optimize vaccine design, the focus was placed on the predicted extracellular regions of the proteins due to their potential surface accessibility. For VacA, only the region encompassing amino acids 58–1290 was selected, excluding putative inner and transmembrane domains predicted by TMHMM webserver. Conversely, the complete sequences of CagA and BabA were chosen as their predicted localization on the external surface of the bacteria (S1 Fig).

### Prediction and screening of B‐cell and T‐cell epitopes

Following the determination of linear B-cell (LBL) epitopes by the ABCpred server, a substantial number of epitopes were identified with scores exceeding the 0.51 threshold. Subsequent filtering of the identified epitopes based on antigenicity, allergenicity, and toxicity criteria yielded 16 epitopes from BabA, 26 epitopes from CagA, and 43 epitopes from VacA, all of which exhibited antigenic properties without displaying allergenic or toxic characteristics (Table 1 in S1 Text).

The MHC I prediction tool on the IEDB website was used to identify CTL epitopes. These epitopes were subsequently filtered based on an antigenicity score exceeding 1.0, alongside the absence of toxic, homologous, and allergenic properties, and a lower IC50 value. Following this screening process, 20 epitopes from the BabA protein, 21 epitopes from the CagA protein, and 34 epitopes from the VacA protein were identified. These epitopes are characterized as antigens, non-allergens, non-toxins, non-homologous, and have an IC50 value below 100 (able 2 in S1 Text).

The article "Immunoinformatic strategy for developing multi-epitope subunit vaccine against Helicobacter pylori" was retracted in 2025. Reasons: compromised peer review; concerns about the authorship.

HTL epitopes were predicted using the MHC II prediction tool on the IEDB website. The identified epitopes were then filtered based on their antigenicity, allergenicity, toxicity, IFN-γ, IL-4, IL-10 production, and lower IC50 value. After removing undesired properties, 13 epitopes from BabA, 2 epitopes from CagA, and 5 epitopes from VacA were identified. These epitopes are immunogenic, do not stimulate any allergic reaction, do not produce any toxins, and have an IC50 value below 50. Additionally, specific HTL epitopes were capable of stimulating the production of IL-4, IL-10, and IFN-γ cytokines, as shown in Table 3 in S1 Text. Among the predicted potential epitopes from BabA, CagA, and VacA, only the top-scoring epitopes chosen for vaccine construction are listed in Table 1.

**Table 1:** Predicted LBL, CTL, and HTL epitopes from BabA, CagA, and VacA proteins for the development of multi-epitope vaccine.

Epitope	Protein	Epitope Sequence	Start Position	Combined Score/ ic50 Value	Antigenicity	Allerginicity	Toxicity	Homology
LBL Epitopes	BabA	CGGNANGQTSTSSTTI	136	0.96	2.1158	Non-allergen	Non-toxin	NH
		GTSGTQGSAPGTVTTQ	436	0.80	1.9923	Non-allergen	Non-toxin	NH
		NNPSTAGTSGTQGSAP	430	0.81	1.8836	Non-allergen	Non-toxin	NH
		EVTGVDKQDNGSKTKT	231	0.86	1.7223	Non-allergen	Non-toxin	NH
		GAELKYRRLYSVYLNY	736	0.79	1.3763	Non-allergen	Non-toxin	NH
	CagA	EKEVAKKLESRNDNKN	626	0.9	1.3551	Non-allergen	Non-toxin	NH
		DVEGVADKDPNYKFNQ	277	0.89	1.3372	Non-allergen	Non-toxin	NH
		RHDWNATVGYKNQQGS	329	0.79	1.3213	Non-allergen	Non-toxin	NH
		NGGPEARHDWNATVGY	323	0.8	1.189	Non-allergen	Non-toxin	NH
		NKKQSSDLKETLNQEP	218	0.82	1.0787	Non-allergen	Non-toxin	NH
	VacA	FVEINNRVGSGAGRKA	143	0.92	1.9154	Non-allergen	Non-toxin	NH
		RVGSGAGRKASSTVLT	149	0.71	1.8981	Non-allergen	Non-toxin	NH
		HYWVKGGQQNKLEVDM	64	0.78	1.3928	Non-allergen	Non-toxin	NH
		KDKPSNTTQNNANNNQ	279	0.88	1.3924	Non-allergen	Non-toxin	NH
		GGYKDKPKDKPSNTTQ	272	0.84	1.2513	Non-allergen	Non-toxin	NH
CTL Epitopes	BabA	AMNGIGIQV	577	7.86	1.9313	Non-allergen	Non-toxin	NH
		GAMNGIGIQV	576	39.85	1.8377	Non-allergen	Non-toxin	NH
		MNVANFQFLF	685	45.39	1.7906	Non-allergen	Non-toxin	NH
		VYLNYVFAY	747	23.43	1.5743	Non-allergen	Non-toxin	NH
		YSVYLNYVF	745	25	1.5447	Non-allergen	Non-toxin	NH
		NFQFLFNMGV	689	30.93	1.5372	Non-allergen	Non-toxin	NH
	CagA	WLDIFLSFVF	208	42.4	1.8438	Non-allergen	Non-toxin	NH
		IFLSFVFNK	211	31.54	1.2369	Non-allergen	Non-toxin	NH
		NFKYTNASK	504	42.68	1.2204	Non-allergen	Non-toxin	NH
		KIGFNQKNMK	1105	48.95	1.0979	Non-allergen	Non-toxin	NH
		WLDIFLSFV	208	15.69	1.062	Non-allergen	Non-toxin	NH
	VacA	AGSSANFEFK	410	23.06	2.1476	Non-allergen	Non-toxin	NH
		NVAVKNFNI	485	81.29	2.1339	Non-allergen	Non-toxin	NH
		RVNNQVGGY	399	14.18	1.5337	Non-allergen	Non-toxin	NH
		TTNAAHLHI	359	48.85	1.4614	Non-allergen	Non-toxin	NH
		EVNFNHLTV	227	35.71	1.2561	Non-allergen	Non-toxin	NH
		TDTKNGTATF	422	99.68	1.348	Non-allergen	Non-toxin	NH
HTL Epitopes	BabA	GAELKYRRLYSVYLN	736	4.6	1.4181	Non-allergen	Non-toxin	NH
		MGAELKYRRLYSVYL	735	7.3	1.2304	Non-allergen	Non-toxin	NH
		AELKYRRLYSVYLNY	737	3.9	1.2255	Non-allergen	Non-toxin	NH
	CagA	EVSYTLKDYGKKQDK	466	8.4	0.8722	Non-allergen	Non-toxin	NH
		DKIVAHNVGSAHLSE	1088	24.7	0.6481	Non-allergen	Non-toxin	NH
	VacA	YHYLAYSAATRASYG	1073	18.7	0.7669	Non-allergen	Non-toxin	NH
		SYHYLAYSAATRASY	1072	3.2	0.5762	Non-allergen	Non-toxin	NH
		QSYHYLAYSAATRAS	1071	4.4	0.5637	Non-allergen	Non-toxin	NH

The article "Immunoinformatic strategy for developing multi-epitope subunit vaccine against Helicobacter pylori" was retracted in 2025. Reasons: compromised peer review; concerns about the authorship.

### Epitopes to HLA alleles molecular docking

Molecular docking performed using the ClusPro web server demonstrated robust interactions between the epitopes derived from BabA, CagA, and VacA proteins and their corresponding HLA alleles (Table 2). The stability of these interactions was further validated by the binding affinity (ΔG) values obtained from the PRODIGY web server. Negative ΔG values, expressed in kcal/mol, are indicative of thermodynamically favorable interactions, with lower ΔG values reflecting stronger binding affinities. These results underscore the stability and suitability of the selected epitopes for eliciting immune responses through HLA-mediated antigen presentation.

**Table 2:** Binding of CTL and HTL epitopes to MHC class I and II alleles.

Type of T Lymphocyte	Epitope	MHC Allele	PDB ID of MHC Allele	ΔG (kcal/mol)
CTL	WLDIFLSFVF	HLA-B*15:01	8ELG	-12.7
	IFLSFVFNK	HLA-A*68:01	6PBH	-12.4
	NFKYTNASK	HLA-A*68:01	6PBH	-12.6
	KIGFNQKNMK	HLA-A*03:01	7MLE	-12.6
	WLDIFLSFV	HLA-A*02:01	7SA2	-12.4
	AMNGIGIQV	HLA-A*02:03	3OX8	-13.1
	GAMNGIGIQV	HLA-A*02:06	3OXR	-13.0
	MNVANFQFLF	HLA-A*68:01	6PBH	-12.3
	VYLNYVFAY	HLA-A*24:02	7SRK	-9.7
	YSVYLNYVF	HLA-B*58:01	7X00	-12.6
	NFQFLFNMGV	HLA-A*02:01	7SA2	-12.6
	AGSSANFEFK	HLA-A*11:01	6ID4	-12.9
	NVAVKNFNI	HLA-A*02:01	7SA2	-12.6
	RVNNQVGGY	HLA-B*15:01	8ELG	-12.6
	TTNAAHLHI	HLA-B*58:01	7X00	-13.2
	EVNFNHLTV	HLA-A*02:03	3OX8	-13.0
	TDTKNGTATF	HLA-B*15:01	8ELG	-13.0
HTL	EVSYTLKDYGKKQDK	HLA-DRB1*15:01	5V4M	-20.7
	DKIVAHNVGSAHLSE	HLA-DRB1*01:01	5V4N	-21.5
	GAELKYRRLYSVYLN	HLA-DRB1*15:01	5V4M	-20.6
	MGAELKYRRLYSVYL	HLA-DRB1*04:01	5JLZ	-21.2
	AELKYRRLYSVYLNY	HLA-DQB1*02:01	4D8P	-25.5
	YHYLAYSAATRASYG	HLA-DRB1*01:01	5V4N	-23.7
	SYHYLAYSAATRASY	HLA-DRB1*01:01	5V4N	-23.5
	QSYHYLAYSAATRAS	HLA-DRB1*01:01	5V4N	-20.8

### Analysis of population coverage

The chosen CTL and HTL epitopes achieved a coverage of 98.55% and 99.99% of the worldwide population, respectively. Notably, when the two types of epitopes were combined, the resulting alleles provided complete coverage of the global population. As illustrated in Fig 2, the epitopes display broad applicability across diverse populations, with only minor variations in effectiveness observed among different ethnic and geographical groups. These results underscore the potential of the selected epitopes to elicit an immune response across a wide demographic, supporting their utility in universal vaccine design.

The article "Immunoinformatic strategy for developing multi-epitope subunit vaccine against Helicobacter pylori" was retracted in 2025. Reasons: compromised peer review; concerns about the authorship.

**Fig 2:** Country-specific population coverage of predicted CTL and HTL epitopes. Population coverage for the epitopes is depicted by bar graphs, presented both collectively and separately for the selected CTL (red bars) and HTL (green bars) epitopes, along with their combined coverage (blue bars). Data indicates that the combined epitopes provide nearly 100% global population coverage, with only minimal variation among regions.

### Vaccine construction and identification of the vaccine properties

Two vaccine designs were developed, each intended to elicit CTL, HTL, and B-cell immune responses by targeting specific epitopes. Each design was further divided into three models based on the selected adjuvants. The adjuvants used to enhance the antigenic response were Melittin, Beta-defensin, and ribosomal protein L7/L12. In total, 12 vaccine constructs were generated by varying the adjuvant type and linker position (S2 Fig).

The immunogenicity, toxicity, and allergenicity of these subunit vaccine candidates were assessed using previously indicated web servers. Vaxijen provided antigenicity scores for all designed constructs, ranging from 0.8467 to 1.1965, indicating that all constructs can stimulate a strong immune response within the body. AllerTOP v.2.0 verified the compatibility of the vaccine candidates, ensuring that no construct would induce allergic reactions. Additionally, all vaccines were found to be non-toxic, meaning they do not cause any toxigenic reactions in the host system.

The aliphatic index for the vaccine constructs in designs 1 and 2 ranged from 62.43 to 80.76, indicating their compatibility with thermostability. A higher aliphatic index suggests greater resistance to temperature fluctuations, underscoring the robustness of the designed vaccines. The instability index of the 12 constructs ranged from 16.52 to 26.42. An instability index lower than 40 signifies the stability of a protein, confirming that all our designed constructs can be considered stable. The GRAVY (Grand Average of Hydropathicity) index values confirmed the hydrophilic nature of the constructs in both designs, highlighting their ability to interact with surrounding water molecules, which is critical for solubility and biological activity. Predictions from the SOLpro server further validated that all the proposed vaccine candidates are soluble, supporting their suitability for further development. Comprehensive data on these analyses is presented in (S1 Table).

The article "Immunoinformatic strategy for developing multi-epitope subunit vaccine against Helicobacter pylori" was retracted in 2025. Reasons: compromised peer review; concerns about the authorship.

### Structural prediction and validation of vaccine constructs

The secondary structure attributes of the vaccine constructs were predicted using the SOPMA tool, which quantified the structural composition of each construct (S2 Table). To determine the tertiary structures of the models, the protein sequences of all twelve were uploaded to the Robetta webserver. The website performed a comprehensive analysis of the protein sequences and produced a probable 3-dimensional configuration for each structure. These initial models were further refined using the GalaxyRefine online tool to enhance their structural quality for subsequent analyses.

To identify the most promising vaccine candidates, the Ramachandran plot was employed. Based on the highest percentage of residues falling within the allowed regions of the plot, one construct from each design (designs 1 and 2) was selected. These constructs were designated as HP_VaX_V1 and HP_VaX_V2, respectively. The structural details of our two final selected constructs are shown in Fig 3. The construct HP_VaX_V1 exhibited a composition of 93.5%, while HP_VaX_V2 demonstrated a composition of 90.4% in the most preferred region (Fig 4). Next, the ProSA web server was utilized to ascertain the Z value of each vaccine design (Fig 5), which indicates the energy distribution of random conformations. Structural assessment revealed that the Z-scores for the first candidate is -5.26 and for the second candidate is -3.64, which is within the normal range for natural protein structures. Additionally, the physicochemical properties of both vaccine candidates were evaluated, and all parameters were found to be within acceptable ranges, supporting their suitability as vaccine candidates (Table 3).

**Fig 3:** 3D structural models and epitope mapping of HP_VaX_V1 and HP_VaX_V2. (a) & (b) 3D structures of both selected vaccines, HP_VaX_V1 and HP_VaX_V2. (c) & (d) Epitope sequences and linker/adjuvant arrangement for HP_VaX_V1 and HP_VaX_V2.

**Fig 4:** Analysis of the Ramachandran plot of HP_VaX_V1 and HP_VaX_V2. (a) HP_VaX_V1 exhibits a 93.5% presence inside the permissible zone, while 5.4% and 0.3% are found in the supplementary and highly permissive regions, respectively. Only 0.8% exhibited presence in the prohibited area. (b) HP_VaX_V2 exhibits a 90.4% presence inside the permissible range, with 6.8% and 1.6% presence in the supplementary and generously permissible regions, respectively. Only 1.2% of the data fell within the prohibited zone.

The article "Immunoinformatic strategy for developing multi-epitope subunit vaccine against Helicobacter pylori" was retracted in 2025. Reasons: compromised peer review; concerns about the authorship.

**Fig 5:** ProSA validation and Z-score analysis of vaccine candidates HP_VaX_V1 and HP_VaX_V2. (a) The Z-score for the ProSA validation of the HP_VaX_V1 vaccine model is –5.26, (b) The Z-score for the ProSA validation of the HP_VaX_V2 vaccine model is –3.64.

**Table 3:** Physicochemical characteristics of vaccine candidates.

Physiochemical properties	Results	
	HP_VaX_V1	HP_VaX_V2
Number of amino acids	733	378
Molecular weight	79841.20	40550.32
Theoretical pI	9.77	9.07
Formula	C_3609_H_5533_N_985_O_1050_S_10_	C_1796_H_2791_N_495_O_563_S_7_
Instability index	19.45	26.48
Aliphatic index	62.43	68.25
Grand average of hydropathicity (GRAVY)	-0.566	-0.489
Estimated half-life (mammalian reticulocytes, *in vitro*)	30 hours	30 hours
Estimated half-life (yeast, *in vivo*)	>20 hours	>20 hours
Estimated half-life (*Escherichia coli*, *in vivo*)	>10 hours	>10 hours
Extinction coefficients (at 280 nm in water)	126410	54780
Antigenicity (Vaxijen)	1.1965	1.0133
Allergenicity (AllerTOP)	Non-Allergen	Non-Allergen
Toxicity	Non-Toxic	Non-Toxic
Solubility (SOLpro)	0.747256	0.832758

### Disulfide modification of the vaccine construct

Using the Disulfide by Design 2.12 server, 79 potential disulfide bond pairs were predicted among the amino acid residues in both vaccine candidates. Based on bond energy values and Chi3 angles, key pairs located within the flexible loop region of the vaccine protein were selected for modification (S3 Table). In the refined tertiary structure, cysteine residues were introduced at positions 188GLY-191ALA and 572ILE-584ALA in HP_VaX_V1, and at 72THR-80ALA in HP_VaX_V2 (S3 Fig). These modifications aimed to stabilize the flexible loop regions and reinforce the structural integrity of the vaccine constructs, thereby improving their thermal stability and functional robustness.

### Conformational B-cell epitope prediction

Conformational B-cell epitopes were predicted using the ElliPro web server, which identifies three-dimensional epitopes capable of stimulating B-cell activation. Analysis of the vaccine constructs revealed that HP_VaX_V1 generated a total of 10 conformational B-cell epitopes (Fig 6), while HP_VaX_V2 exhibited 6 epitopes (Fig 7). These findings highlight the potential of both constructs to elicit robust humoral immune responses (S4 Table).

**Fig 6:** B-cell epitope predictions for HP_VaX_V1. The purple regions illustrate the epitopes as identified by the ElliPro webserver, along with their respective length and score listed below.

**Fig 7:** B-cell epitope predictions for HP_VaX_V2. The yellow regions illustrate the epitopes as identified by the ElliPro webserver, along with their respective length and score listed below.

The article "Immunoinformatic strategy for developing multi-epitope subunit vaccine against Helicobacter pylori" was retracted in 2025. Reasons: compromised peer review; concerns about the authorship.

### Molecular docking of HP_VaX_V1 and HP_VaX_V2

A docking analysis was conducted using ClusPro to investigate the molecular interaction between the vaccine constructs and potential Toll-Like Receptors (TLRs). Eight Toll-like receptors (TLRs), including TLR2, TLR3, TLR4, TLR5, TLR6, TLR7, TLR8, and TLR9, were chosen as potential targets due to their role in recognizing and initiating immune responses against pathogen (Fig 8). Binding affinities were determined using the PRODIGY platform based on negative ΔG values, which represent the change in Gibbs free energy during binding. Negative ΔG values indicate thermodynamically favorable interactions, with lower values signifying stronger and more stable binding [52]. This is particularly relevant in vaccine design, as strong binding between vaccine constructs and TLRs suggests a greater potential to elicit robust immune responses. HP_VaX_V1 exhibited the strongest affinity toward TLR7 (ΔG = −20.3 kcal/mol, Kd (M) at 25.0°C), whereas HP_VaX_V2 exhibited a greater preference for TLR8 (ΔG = −20.9 kcal/mol, Kd (M) at 25.0°C). As a result, the high binding affinity of these two constructs (HP_VaX_V1 and HP_VaX_V2) with their respective TLRs prioritized their further investigation. The PDBsum analysis provided a comprehensive elucidation of the precise interactions between the residues of the vaccine constructs and Toll-like receptors (TLRs). Specifically, HP_VaX_V1 formed 6 salt bridges, 20 hydrogen bonds, and 255 non-bonded contacts, while HP_VaX_V2 established 6 salt bridges, 37 hydrogen bonds, and 314 non-bonded contacts (Fig 9).

**Fig 8:** Molecular docking analysis of HP_VaX_V1 and HP_VaX_V2 with Toll-Like Receptors (TLRs). Binding conformations of HP_VaX_V1 (blue) and HP_VaX_V2 (red) with eight Toll-Like Receptors (TLRs), including TLR2, TLR3, TLR4, TLR5, TLR6, TLR7, TLR8, and TLR9. The ΔG values (in kcal/mol) below each structure represent the binding affinities, with more negative values indicating stronger and more stable interactions.

**Fig 9:** Comparative interaction network analysis of HP_VaX_V1 and HP_VaX_V2 with TLR7 and TLR8. Detailed interaction networks between HP_VaX_V1 and TLR7 (left panel), and HP_VaX_V2 and TLR8 (right panel). The interactions include salt bridges, disulfide bonds, hydrogen bonds, and non-bonded contacts, visualized as connections between amino acid residues from the vaccine constructs and Toll-Like Receptors. Each interaction type is represented by a specific color-coded line, as indicated in the key below.

The article "Immunoinformatic strategy for developing multi-epitope subunit vaccine against Helicobacter pylori" was retracted in 2025. Reasons: compromised peer review; concerns about the authorship.

### Normal mode analysis

A Normal Mode Analysis (NMA) was performed using the iMODS web server to assess the stability and adaptability of the Human TLR-Vaccine construct. The iMODS server successfully predicted numerous dynamic states of the vaccine candidates with high precision. The analysis focused on the HP_VaX_V1-TLR7 and HP_VaX_V2-TLR8 complexes due to their strongest binding affinities for their respective toll-like receptors, as determined by the PRODIGY webserver (Fig 10). The deformability profiles of both constructs indicate overall low deformability with some localized peaks, suggesting rigidity in most regions and flexibility in non-critical areas (Fig 10A). The B-factors from NMA closely align with the experimental PDB B-factors for both constructs, with only minor deviations, supporting the reliability and stability of the modeled structures (Fig 10B). Both constructs exhibit low first eigenvalues (4.580659e-06 and 3.543521e-06, respectively), indicating minimal energy is required for their primary modes of motion, which is a positive indicator of stability (Fig 10C). The cumulative variance explained by the first 20 modes is substantial for both constructs, demonstrating that the essential motions are well captured (Fig 10D). Covariance maps for both constructs show a balanced mix of correlated and anti-correlated movements, indicating stable structures with defined dynamic regions (Fig 10E). Additionally, the elastic network models reveal strong interactions in key regions, further suggesting structural rigidity (Fig 10F). Overall, both vaccine constructs demonstrate characteristics of stable structures according to the iMODS analysis, indicating their potential efficacy and reliability.

**Fig 10:** Molecular dynamic simulation of the HP_VaX_V1-TLR7 and HP_VaX_V2-TLR8 constructs. (a) Deformability of the protein structures, illustrating the flexibility at each residue. (b) B-factor (or temperature factor) analysis, showing the degree of atomic displacement. (c) Eigenvalues from the Normal Mode Analysis (NMA), indicating the stiffness of the modes. (d) Variance map, representing the contribution of each mode to the overall motion. (e) Co-variance map, highlighting correlated motions between residues. (f) Elastic network model, depicting the connections and interactions within the protein structure.

### Molecular dynamics simulation analyses

MD simulation provides crucial insights into the dynamic behavior, structural stability, and flexibility of biomolecular systems under physiological conditions. In the context of drug or vaccine design, MD simulations provide a deeper evaluation of molecular interactions, stability, and conformational changes in protein complexes, complementing static structural analyses such as molecular docking [88, 89]. In this study, 100 ns MD simulations were performed to analyze the dynamic properties of the HP_VaX_V1-TLR7 and HP_VaX_V2-TLR8 complexes. Key parameters such as Root Mean Square Deviation (RMSD), Root Mean Square Fluctuation (RMSF), Radius of Gyration (Rg), Principal Component Analysis (PCA), and Free Energy Landscape (FEL) were systematically assessed.

The article "Immunoinformatic strategy for developing multi-epitope subunit vaccine against Helicobacter pylori" was retracted in 2025. Reasons: compromised peer review; concerns about the authorship.

#### Root Mean Square Deviation (RMSD) analysis

The Root Mean Square Deviation (RMSD) measures the average deviation of atomic positions of a biomolecular complex from a reference structure over time. It is a fundamental parameter in molecular dynamics simulations to evaluate the structural stability and convergence of the system [90–92]. The RMSD plots of the HP_VaX_V1-TLR7 and HP_VaX_V2-TLR8 complexes during the 100 ns simulation are depicted in Fig 11A. For HP_VaX_V1-TLR7, the RMSD values started at approximately 2 Å and showed an initial increase, stabilizing around 10 Å after 20 ns. As the simulation progressed, minor fluctuations were observed, with values peaking around 25 Å before settling at approximately 20 Å during the latter stages. Similarly, HP_VaX_V2-TLR8 exhibited RMSD values starting at 2 Å and stabilizing around 5–10 Å after 20 ns. The trajectory remained steady throughout the simulation, with minimal fluctuations observed, indicating strong structural consistency and adaptability under simulated conditions. These results affirm that both HP_VaX_V1-TLR7 and HP_VaX_V2-TLR8 maintain their structural stability during molecular dynamics simulations, reflecting their robustness and quality as vaccine constructs.

**Fig 11:** Structural stability and residue flexibility analyses of the HP_VaX_V1-TLR7 and HP_VaX_V2-TLR8 protein complexes over a 100 ns MD simulation. (A) Root Mean Square Deviation (RMSD) plot illustrating the structural stability of HP_VaX_V1-TLR7 (black) and HP_VaX_V2-TLR8 (red) complexes. (B) Root Mean Square Fluctuation (RMSF) plot showing the residue-wise flexibility of HP_VaX_V1-TLR7 (black) and HP_VaX_V2-TLR8 (red).

#### Root Mean Square Fluctuation (RMSF) analysis

The Root Mean Square Fluctuation (RMSF) provides insights into the local flexibility of individual residues in the protein-protein complexes. It quantifies the deviation of atomic positions from their average, thus highlighting the regions that exhibit dynamic behavior [93–96]. The RMSF analysis of the HP_VaX_V1-TLR7 and HP_VaX_V2-TLR8 complexes, as shown in Fig 11B, revealed favorable structural integrity, with low RMSF values across most residues, indicating a stable core structure and limited atomic fluctuations. Peaks in RMSF were observed primarily in terminal and loop regions, which are inherently more flexible. Key residues exhibiting notable fluctuations included HSD188, MET189, THR190, ASP38, LEU39, LYS75, ASP76, GLU77, THR270, ASN271, VAL272, and LYS273, with LYS273 at the N-terminal displaying the highest RMSF values, exceeding 50 Å in both constructs. In the HP_VaX_V1-TLR7 complex, occasional peaks reached approximately 20 Å around atom indices 5,000 and above 50 Å near atom index 10,000, while the HP_VaX_V2-TLR8 complex exhibited a similar pattern with terminal fluctuations slightly exceeding 50 Å. These results highlight the stability and structural integrity of both vaccine constructs, with localized flexibility supporting effective molecular interactions, further validating their potential as robust vaccine candidates.

The article "Immunoinformatic strategy for developing multi-epitope subunit vaccine against Helicobacter pylori" was retracted in 2025. Reasons: compromised peer review; concerns about the authorship.

#### Radius of Gyration (Rg) analysis

The Radius of Gyration (Rg) is a parameter that measures the compactness of a biomolecular structure by calculating the distribution of its atomic mass around the center of mass. The Rg values provide insights into the spatial distribution of atoms around the center of mass of the molecule over the simulation time [81, 97]. As shown in Fig 12A, the Rg profiles of both vaccine constructs, HP_VaX_V1 (black line) and HP_VaX_V2 (red line), were monitored throughout the 100 ns simulation period. Both constructs exhibited consistent Rg values without significant fluctuations, indicating structural compactness and stability under simulated physiological conditions. Specifically, HP_VaX_V1 maintained an average Rg value of approximately 3.2–3.4 Å, while HP_VaX_V2 exhibited a slightly higher average Rg value of around 3.5–3.7 Å. These stable Rg trends suggest that both vaccine constructs have well-folded structures with no evidence of unfolding or structural destabilization. These observed stability and compactness reflect the high-quality design of both constructs, which were optimized for antigenicity and structural integrity during the vaccine design process.

**Fig 12:** Compactness and conformational stability analysis of vaccine constructs. (A) Radius of Gyration (Rg) plot depicting the compactness of HP_VaX_V1 (black) and HP_VaX_V2 (red) over a 100 ns molecular dynamics simulation. (B) Principal Component Analysis (PCA) scatter plot illustrating the conformational stability of HP_VaX_V1 (black) and HP_VaX_V2 (red) by projecting their molecular dynamics trajectories onto principal eigenvectors.

#### Principal Component Analysis (PCA)

To assess the dynamic behavior and stability of the vaccine constructs HP_VaX_V1 and HP_VaX_V2, principal component analysis (PCA) was performed. PCA evaluates the collective motion of the constructs by projecting their trajectories onto principal eigenvectors [89, 98]. The resulting PCA scatter plots are shown in Fig 12B. Both vaccine constructs exhibited restricted and compact projections on the PCA plane, indicating their conformational stability and structural quality. The clustering patterns observed in the projections suggest that the vaccine constructs maintained stable conformations throughout the simulations. Specifically, HP_VaX_V1 demonstrated tightly packed projections along the principal eigenvectors, reflecting minimal large-scale structural fluctuations. Similarly, HP_VaX_V2 showed consistent and stable clustering, further confirming its structural integrity under simulated conditions. These results establish that both vaccine constructs are of high quality and maintain robust conformational stability, making them strong candidates for further validation.

The article "Immunoinformatic strategy for developing multi-epitope subunit vaccine against Helicobacter pylori" was retracted in 2025. Reasons: compromised peer review; concerns about the authorship.

#### Free Energy Landscape (FEL) analysis

The Free Energy Landscape (FEL) provides a thermodynamic perspective of the system’s conformational stability. FEL maps are constructed based on the principal components, with low-energy regions corresponding to stable conformational states and high-energy regions indicating less favorable, unstable states. These landscapes visually represent the system’s propensity to occupy specific conformations over the simulation time [99]. For both complexes, the FELs were constructed by mapping the first two principal components (PC1 and PC2) against their corresponding Gibbs free energy values (Fig 13). The FEL map of HP_VaX_V1 exhibits two prominent and deep energy basins, indicating the presence of well-defined, energetically favorable conformational states. The deeper and more compact basins suggest minimal structural fluctuations and high stability throughout the simulation, with a steep energy gradient reflecting limited transitions between states, further implying a highly stable construct. Similarly, the FEL map of HP_VaX_V2 reveals a significant energy basin, though with slightly broader energy regions compared to HP_VaX_V1. The well-defined single deep basin suggests a stable conformational state with limited structural deviations during the simulation, and smooth transitions between low-energy regions highlight the robustness of HP_VaX_V2’s structural stability. Both constructs exhibit clear, deep, and well-distributed basins in the FEL maps, indicating their occupation of energetically favorable and stable conformational states. The lack of scattered or high-energy regions confirms that neither construct undergoes significant structural deviations, ensuring consistent stability throughout the molecular dynamics simulations. Additionally, the smoothness of the energy landscapes and clustering of low-energy conformations further support the high structural quality of both vaccine constructs, reinforcing their potential for immunogenic effectiveness.

The article "Immunoinformatic strategy for developing multi-epitope subunit vaccine against Helicobacter pylori" was retracted in 2025. Reasons: compromised peer review; concerns about the authorship.

**Fig 13:** Free Energy Landscape (FEL) analysis of vaccine constructs. (A) FEL map of HP_VaX_V1 constructed using the first two principal components (PC1 and PC2). The map reveals two prominent and deep energy basins, representing highly stable and energetically favorable conformational states. (B) FEL map of HP_VaX_V2 constructed using the same parameters. The map exhibits a well-defined single deep energy basin, suggesting a stable conformational state with limited structural deviations.

### Immune simulation

The C-ImmSim server was used to mimic the immunological response elicited by the developed HP_VaX_V1 and HP_VaX_V2 vaccines. The simulation results, presented in Fig 14, demonstrate the primary and secondary immune responses of the host to the vaccine candidates. Each vaccine administration resulted in a notable rise in antigen levels, which subsequently decreased over time, accompanied by a pronounced surge in immunoglobulin levels. The rapid initial rise in IgG and IgA concentrations suggests a strong humoral response, with IgG1 and IgA1 dominating early. The gradual decline after the peak indicates that antibody levels taper off, reflecting the waning of the humoral memory over time. The simulation indicated that the elevated levels of specific IgG isotypes persisted longer than IgM, suggesting the establishment of durable humoral memory. Additionally, the coordinated rise in cytotoxic T-cells (Tc) alongside the humoral response highlights a balanced activation of both arms of the immune system, essential for robust and long-lasting protection against future infections (Fig 14A). The B-cell population dynamics revealed significant changes in the B-cell population, with the emergence of multiple B-cell isotypes. This indicates robust adaptive immunity, including the formation of memory B cells and evidence of class switching. Memory B cells demonstrated persistence over time, enabling long-term humoral immunity even as effector B cells declined (Fig 14B). The dendritic cell (DC) population displayed consistent activity throughout the simulation, emphasizing their role in antigen presentation and T-cell activation. Various states of DCs were observed, with presenting dendritic cells maintaining steady levels, indicating continuous antigen presentation that supports prolonged cell-mediated immune responses (Fig 14C). Helper T-cell (Th) responses exhibited an initial sharp increase in active Th cells immediately post-vaccination, followed by a transition to a higher population of resting Th cells, indicative of immune memory formation (Fig 14D). The Th cell population dynamics highlight the shift from an effector state to a memory state, ensuring sustained immune readiness for future antigenic challenges. Similarly, the cytotoxic T-cell (Tc) population also demonstrated a rapid rise in active Tc cells post-vaccination, followed by a decline and an increase in resting Tc cells, signifying the establishment of long-term immune memory. This balance between active and resting Tc cells indicates a robust yet transient cytotoxic response, with sustained immune surveillance through memory Tc cells (Fig 14E). Additionally, the levels of interferon-gamma (IFN-γ) spiked following the second vaccine dose, reflecting a strong Th1-type immune response. The low Simpson index (D) indicated a diverse T-cell receptor (TCR) repertoire, underscoring the effectiveness of the immune response. The rise and subsequent decline in active Tc cells further demonstrated a transient but potent cytotoxic response, with memory Tc cells persisting to provide long-term immune surveillance (Fig 14F). Overall, the *in silico* immune simulation demonstrated that both HP_VaX_V1 and HP_VaX_V2 vaccines successfully induced a strong and durable immune response, characterized by the growth of various immune cell types and the generation of memory cells.

The article "Immunoinformatic strategy for developing multi-epitope subunit vaccine against Helicobacter pylori" was retracted in 2025. Reasons: compromised peer review; concerns about the authorship.

**Fig 14:** Immune simulation results for HP_VaX_V1 and HP_VaX_V2 vaccine constructs. (a) The black line represents antigen levels, signifying the production of immunoglobulin after immunization. (b) The B-cell population dynamics after multiple encounters with the antigen. (c) The dendritic cell population at various stages over a one-year period post-initial injection. (d) The Simpson index quantifies the interferon-gamma response within one year post-immunization. (e) The data for the population of Helper T-cells. (f) The concentration of Cytotoxic T-cells assessed over a one-year period after the initial antigen encounter.

### *In Silico* expression prediction and cloning of HP_VaX_V1 and HP_VaX_V2

The codon-optimized sequences for HP_VaX_V1 and HP_VaX_V2 exhibited high codon adaptation index (CAI) values of 0.92 and 0.93, respectively, indicating a strong likelihood of successful expression within the bacterial system. This value is very close to the ideal value of 1.0, indicating optimal codon usage. Furthermore, the GC content for both vaccine candidates was calculated as 52.11% and 52.82%, which falls within the preferred range of 30% to 70% for *E*. *coli* expression. The codon frequency distribution (CFD) analysis indicated no unusual consecutive codons (0%) within the optimized sequence. The presence of such tandem rare codons can negatively impact translation rate or or completely stop the translation process. The vaccine mRNA’s stability was verified by the negative free energy values of -760.60 kcal/mol and -411.70 kcal/mol for HP_VaX_V1 and HP_VaX_V2, respectively, as calculated by the RNAfold tool (Fig 15). Finally, using the SnapGene program, the optimized vaccination sequences were incorporated into the pET28a(+) expression vector to facilitate expression. This insertion occurred between the Eco53KI and BstZ17I restriction sites. The cloned HP_VaX_V1 and HP_VaX_V2 constructs, which contained the recombinant plasmid, were determined to be 4755 bp and 3609 bp in length, respectively (Fig 16).

The article "Immunoinformatic strategy for developing multi-epitope subunit vaccine against Helicobacter pylori" was retracted in 2025. Reasons: compromised peer review; concerns about the authorship.

**Fig 15:** Computational predictions of secondary structures for HP_VaX_V1 and HP_VaX_V2 mRNAs. Predicted minimum free energy (MFE) secondary structures of (A) HP_VaX_V1 mRNA (-760.60 kcal/mol) and (B) HP_VaX_V2 mRNA (-411.70 kcal/mol). Base pairs are represented by lines, with color gradients indicating base pairing probability.

**Fig 16:** Schematic representation of recombinant expression plasmids for HP_VaX_V1 and HP_VaX_V2. Circular maps of the pET-28a(+) expression vectors harboring the (a) HP_VaX_V1 and (b) HP_VaX_V2 gene inserts. Key features include the multiple cloning site (MCS), antibiotic resistance gene, origin of replication (ori), and T7 promoter. Restriction enzyme sites are indicated.

## Discussion

*Helicobacter pylori* infection is a significant public health concern because there is presently no approved vaccine or effective treatment for this infection. This bacterium is responsible for causing several gastrointestinal problems, including peptic ulcers and stomach cancer, highlighting the necessity for a highly efficient vaccine. Despite three decades of research, no putative *H*. *pylori* vaccine has been commercialized, and most documented clinical trials have concluded at phase I [100]. In response to this unmet medical need, immunoinformatics analyses were employed to create potential subunit vaccine candidates targeting *H*. *pylori’*s virulent proteins. Traditional vaccine design often focuses on creating a vaccine from a single protein. This approach can be limiting because pathogens can mutate and evade the immune response. To overcome this challenge, our approach involves designing a multi-epitope-based subunit vaccine targeting three essential virulent proteins of *H*. *pylori*: CagA, VacA, and BabA. This strategy aims to elicit a robust and broad immunogenic response, protecting against a wide range of *H*. *pylori* strains. By targeting multiple antigens, the vaccine reduces the likelihood of escape mutations compared to single-antigen vaccines [101, 102]. Additionally, this vaccination approach has demonstrated increased safety and logistical feasibility [103].

The article "Immunoinformatic strategy for developing multi-epitope subunit vaccine against Helicobacter pylori" was retracted in 2025. Reasons: compromised peer review; concerns about the authorship.

To commence this investigation, all possible virulence factors of *H*. *pylori* were studied, and three proteins (BabA, CagA & VacA) were selected based on their critical roles in the pathogenesis and immune evasion strategies of *H*. *pylori*. The CagA protein is a well-known virulence factor that disrupts cellular processes once injected into host cells and induces inflammation, making it a prime target for eliciting a robust immune response [104]. VacA, another major virulence factor, can induce vacuole formation in host cells, suppress immune responses, and promote bacterial survival [105]. Its inclusion in the vaccine design aims to neutralize these effects and improve the overall ability of the vaccination to stimulate an immune response. BabA, an essential adhesin, enables *H*. *pylori* to adhere more easily to the gastric epithelium, which is a necessary process for colonization and long-term survival within the host. Targeting BabA in the vaccine design is intended to prevent the initial stages of infection, thereby reducing bacterial colonization and subsequent pathogenesis [106]. Recent studies have also emphasized the significance of these proteins in triggering robust humoral and cellular immune responses [107–109]. For instance, the immunogenic properties of CagA and VacA have been well-documented, with both proteins showing significant roles in impairing gastric epithelial cell functions [110]. Research by Gordon (2000) demonstrated significant associations between BabA, CagA, and VacA. All patients with duodenal ulcers tested positive for all three markers, while 74% of gastric cancer patients, 35% of MALT lymphoma patients, and 43% of antral gastritis patients were positive for these markers. [30].

Multiple servers were utilized to identify B-cell, CTL, and HTL epitopes for BabA, CagA, and VacA proteins. The epitopes were assessed to determine their antigenicity, allergenicity, homology, and toxicity. Moreover, HTL epitopes capable of eliciting cytokines, including IL-4, IL-10, and interferon-gamma (IFN-γ), were selected. Cytokines serve as essential agents in the body’s defense mechanisms. The CTL and HTL epitopes were further validated through molecular docking with their corresponding MHC-I and MHC-II alleles, revealing strong binding affinities characterized by low ΔG scores (Table 2). These findings indicate a high potential for the predicted epitopes to elicit a robust immunological response. Additionally, the predicted epitopes demonstrated 100% global population coverage, underscoring their broad applicability in diverse populations.

The article "Immunoinformatic strategy for developing multi-epitope subunit vaccine against Helicobacter pylori" was retracted in 2025. Reasons: compromised peer review; concerns about the authorship.

Two distinct design strategies were implemented to assess the potential immunogenicity of the chosen epitopes. Design-1 incorporated short linker sequences between the epitopes. These linkers were designed to minimize potential junctional immunogenicity, a phenomenon where the immune system reacts against the artificial connections between epitopes in a vaccine construct. In contrast, Design-2 adopted a novel vaccine design strategy. This approach incorporated the natural junctional regions between the chosen antigens into the vaccine construct. This approach was intended to potentially induce a more effective and realistic immunological response. In order to increase the ability of the vaccine designs to provoke an immune response, adjuvants were incorporated into both Design-1 and Design-2. By employing three distinct adjuvants (Melittin, β defensin, and Ribosomal protein L7/L12) and altering the arrangement of linker positions in different models, twelve vaccine sequences were developed for subsequent evaluation.

The antigenicity, allergenicity, and physicochemical characteristics of the developed vaccine candidates were analyzed using various computational tools. Solubility, a crucial factor for *in vivo* administration, was also evaluated since insoluble proteins can lead to inconsistencies in vaccine content. The physicochemical analysis indicated the potential thermostability of the selected candidates. Both secondary and tertiary structures were analyzed to evaluate the structural stability of the vaccine candidates. The analysis of secondary structure showed that most models had a high proportion of coil regions. While coils contribute to flexibility, their abundance could impact overall protein structure. To gain further insights into the three-dimensional (3D) conformation, a webserver utilizing a combination of homology modeling and de novo (ab initio) methods was employed. Encouragingly, all vaccine candidates exhibited satisfactory results in the tertiary structure analysis, suggesting their potential suitability for further investigation.

Ramachandran plots were employed to shortlist the most promising vaccine candidates by analyzing the stereochemical properties of the protein residues. Two models exhibited the highest percentage of residues within the allowed regions and were selected as the final vaccine candidates: HP_VaX_V1 and HP_VaX_V2. HP_VaX_V1 exhibited 93.5% of its residues within the allowed region, while HP_VaX_V2 showed 90.4%. Both candidates displayed minimal presence in the disfavored areas. Furthermore, structure validation using Z-scores demonstrated acceptable overall protein structures for both candidates, with Z-scores of -5.26 and -3.64 for HP_VaX_V1 and HP_VaX_V2, respectively. These results suggest that the selected vaccine candidates possess well-defined and structurally sound conformations. Since the three-dimensional (3D) structure brings different protein regions into spatial proximity, these closely associated segments can act as conformational epitopes, triggering B-cell responses. Our candidates, HP_VaX_V1 and HP_VaX_V2, were found to possess ten and six conformational epitopes, respectively.

The article "Immunoinformatic strategy for developing multi-epitope subunit vaccine against Helicobacter pylori" was retracted in 2025. Reasons: compromised peer review; concerns about the authorship.

To assess the potential immunomodulatory effects of the vaccine candidates, molecular docking simulations were conducted to investigate their binding interactions with different Toll-like receptors (TLRs). The binding affinity of each docked complex was estimated by analyzing their negative free energy change (ΔG) values. HP_VaX_V1 and HP_VaX_V2 exhibited the strongest binding affinity with TLR7 & TLR8, with ΔG values of -20.3 kcal/mol and -20.9 kcal/mol, respectively. The intermolecular protein-protein interactions between vaccines and TLRs exhibited numerous salt bridges, hydrogen bonds, and non-bonded contacts, suggesting robust biomolecular stability.

The molecular dynamics simulation (MDS) performed in this study offers significant insights into the structural stability, flexibility, and conformational dynamics of the analyzed protein-protein complex under physiological conditions. The comprehensive analyses, encompassing Root Mean Square Deviation (RMSD), Root Mean Square Fluctuation (RMSF), Radius of Gyration (Rg), Principal Component Analysis (PCA), and Free Energy Landscape (FEL), collectively confirm the robustness and reliability of the modeled complex over the 100 ns simulation timeframe. The RMSD trajectory demonstrated an initial equilibration phase followed by convergence to a stable configuration, indicative of the structural stability of the complex throughout the simulation. This observation is consistent with previously reported findings, where RMSD has been utilized as a reliable metric for assessing protein stability *in silico* [91–93]. Additionally, RMSF analysis revealed localized flexibility, predominantly within terminal and loop regions, which is characteristic of dynamic protein segments involved in molecular interactions. These results align with prior studies, underscoring the functional relevance of such fluctuations in protein complexes [94, 95]. The compactness of the complex, as indicated by the Rg profile, remained stable with minor fluctuations reflective of transient conformational adjustments. Similar trends have been reported in comparable molecular systems, where Rg serves as a critical measure of structural compactness and stability [81, 97]. The PCA further highlighted restricted large-scale motions, with tightly clustered conformations supporting the notion of structural rigidity and stability. Furthermore, the FEL analysis identified distinct low-energy basins, suggesting that the complex predominantly occupies energetically favorable conformations. This observation is consistent with studies that have utilized FEL to validate the thermodynamic stability of protein-protein complexes [99].

The article "Immunoinformatic strategy for developing multi-epitope subunit vaccine against Helicobacter pylori" was retracted in 2025. Reasons: compromised peer review; concerns about the authorship.

Normal mode analysis (NMA) provided additional insights into the stability of the complex. Co-variance plots revealed strong correlations among residues at the binding interfaces, suggesting coordinated movements that contribute to stability.

An *in silico* immune simulation was conducted to forecast the potential immune reaction triggered by the vaccine candidates following administration. This simulation revealed a robust antibody response in both HP_VaX_V1 and HP_VaX_V2 over a one-year timeframe post-vaccination. Following each immunization, B-cell and helper T-cell levels exhibited an initial rise, followed by a gradual decline over time. These decreases coincided with the formation of memory B-cells and resting helper T-cells, suggesting the acquisition of long-term immunological memory. Interestingly, active cytotoxic T-cell (CTL) levels remained consistent throughout the three immunizations, with a subsequent decrease in active cells over time. However, this decrease was accompanied by the formation of resting CTLs, further contributing to the development of immunological memory. Finally, the simulation predicted an increase in cytokine levels with each vaccination, followed by a gradual decrease, reflecting the dynamic nature of the immune response.

To achieve optimal expression levels when delivered via a vector system, the vaccine candidates HP_VaX_V1 and HP_VaX_V2 were codon optimized. Codon adaptation index (0.92 and 0.93) and GC content (52.11% and 52.82%) were assessed for both HP_VaX_V1 and HP_VaX_V2, respectively. These measures suggest that the conditions are ideal for generating a high degree of protein production in *E*. *coli*. Additionally, both constructs were confirmed to be thermostable, as evidenced by their vaccine mRNA having negative free energy values of -760.60 kcal/mol and -411.70 kcal/mol, respectively. Finally, *in silico* molecular cloning was performed to ensure the construct was ready for downstream processing. The *E*. *coli* expression system was chosen for its efficiency in producing large quantities of recombinant protein [111]. The *in silico* cloning successfully ligated both sequences (HP_VaX_V1 and HP_VaX_V2) into the pET28a (+) expression vector, demonstrating that our construct is ready for further experimental validation.

The article "Immunoinformatic strategy for developing multi-epitope subunit vaccine against Helicobacter pylori" was retracted in 2025. Reasons: compromised peer review; concerns about the authorship.

In recent years, researchers have explored the development of multi-epitope vaccines by targeting various bacterial antigens that are capable of eliciting a more robust immunogenic reaction [112–114]. However, many of the multi-epitope-based vaccines were built by focusing on single antigens [115, 116], which could be more susceptible to reduced efficacy due to antigenic variation and mutations. In contrast, our research takes a more robust approach by incorporating epitopes from multiple proteins, specifically CagA, VacA, and BabA. This approach reduces the likelihood that mutations in a single protein will enable the bacterium to escape immune detection. By targeting multiple proteins, our vaccine constructs ensure the immune system can recognize and respond to several antigens, enhancing overall vaccine effectiveness.

Several multi-epitope vaccine candidates have been proposed for *H*. *pylori*, but our study has greater significance compared to most of them. Our analysis predicted high antigenicity levels for both constructs, with scores significantly higher than those reported by Ru et al. (2022) [117], Khan et al. (2019) [118], Urrutia-Baca et al. (2019) [119], and Chaleshtori et al. (2023) [120], indicating a more significant antigenic potential. The *in silico* analysis also revealed a high level of stability for both design models, with an instability index of 19.45 and 26.48, respectively. These values are notably lower compared to those observed in previous research by Ru et al. (2022) [117], Urrutia-Baca et al. (2019) [119], Chaleshtori et al. (2023) [120], and Keshri et al. (2023) [121]. Improved stability reduces the risk of degradation during storage and delivery, ultimately enhancing vaccine efficacy. Additionally, the solubility of our vaccine candidate was determined to be 0.747256 and 0.832758, which are higher values than the results of Shojaeian et al. (2023) [122] and Ghosh et al. (2021) [123]. Enhanced solubility facilitates efficient expression, purification, and formulation of the vaccine, which are crucial steps for successful vaccine development. These qualities collectively suggest that our vaccine constructs are ideal candidates for further research and development. However, the study has limitations, including the lack of experimental validation, the need for long-term immunogenicity studies, and potential challenges with large-scale production in *E*. *coli*. Future steps involve *in vitro* and *in vivo* validation, followed by clinical trials to assess safety, efficacy, and long-term immunity. Optimization for large-scale production and exploration of alternative expression systems will also be critical to ensure accessibility and effectiveness. While challenges remain, this construct represents a significant step forward in developing an affordable and effective vaccine against *H*. *pylori*-associated diseases.

The article "Immunoinformatic strategy for developing multi-epitope subunit vaccine against Helicobacter pylori" was retracted in 2025. Reasons: compromised peer review; concerns about the authorship.

## Conclusions

The development of a safe and effective vaccine against *H*. *pylori* is crucial due to the bacterium’s pathogenic potential, its association with severe gastrointestinal diseases, and the absence of approved therapeutic options. This study employed computational methods to design multi-epitope subunit vaccines that can stimulate a robust immune response encompassing both humoral and cellular immunity. The vaccine designs satisfactorily fulfilled the criteria for antigenicity, allergenicity, immunogenicity, and physicochemical qualities. Three-dimensional structural analysis showed a significant binding affinity between the vaccine constructs and Toll-like receptors, indicating their ability to stimulate both humoral cellular immunological responses. While *in silico* findings suggest a potential immunogenic response, further *in vitro* and *in vivo* assessments are required to establish the vaccine’s efficacy, immunogenicity, and, most importantly, its safety profile prior to human administration.

## Supporting information

S1 Text Prediction of all predicted epitopes from BabA, CagA & VacA. (DOCX)

S1 Fig Surface availability of selected protein candidates. (DOCX)

S2 Fig Epitope mapping of the 12 vaccine models from 2 design groups. (DOCX)

S3 Fig Disulfide engineering in vaccine constructs. (DOCX)

S1 Table Different property analysis of designed vaccine candidates. (DOCX)

S2 Table Predicted secondary and tertiary structure properties of designed vaccine candidates. (DOCX)

S3 Table Predicted disulfide bond partners by disulfide by design 2.0. (DOCX)

S4 Table Predicted discontinuous epitope(s) for HP_VaX_V1 & HP_VaX_V2. (DOCX)
